RETRACTED

# Influence of Underground Mining Direction Based on Particle Flow on Deformation and Failure of Loess Gully Area

**DOI:** 10.1155/2022/1698220

**Published:** 2022-05-13

**Authors:** Yanjun Zhang, Jiayuan Kong, Yuanhao Zhu, Wenxin Zhu, Fushuai He, Lingfei Wang, Zoujun Li

**Affiliations:** ^1^College of Geoscience and Surveying Engineering, China University of Mining and Technology-Beijing, Beijing 100083, China; ^2^School of Mining Engineering, Taiyuan University of Technology, Taiyuan 030024, China; ^3^Power China Zhongnan Engineering Corporation Limited, Changsha 410000, China; ^4^Statistics Bureau of Xinzhou City, Xinzhou 034000, China; ^5^China Energy Engineering Group Shanxi Electric Power Engineering Co., Ltd., Taiyuan 030024, China

## Abstract

Due to unique landform and lithological features of the loess gully area, the geological disasters caused by coal mining have become more complex. Moreover, the advancing direction of the working face has an important influence on the deformation of the slope on both sides of the gully. In this paper, combined with the specific conditions of a coal mine working face in western China, we use the method of particle flow numerical simulation and theoretical analysis to examine and observe the deformation, as well as characteristics of failures in the loess gully area under different mining directions of the working face. The deformation process of the gully area can be obtained by combining the numerical simulation results. According to different mining directions of the working face, the failure mode of mining in the loess gully area was divided into the back slope and along slope advancing failure modes. Through empirical evaluation, our investigation demonstrates that the bottom of the gully was damaged seriously by both along slope mining and back slope mining. Albeit the influence of coal seam excavation on the slope surface was relatively small; however, it is greater on the flat ground of the upper slope. Under the same mining conditions, the advancing direction of the working face affected the horizontal movement of the loess gully area but had less effect on the subsidence. Furthermore, we observed that the failure mode of the mining slope is highly correlated with the mining direction and relative position of the working face. The results obtained from this research can provide useful information for deformation and failure prediction, working face mining method, and geological disaster assessment in the loess gully area.

## 1. Introduction

The Loess gully area is mainly distributed in the Loess Plateau of China, which is a typical landform in the central and western areas [1]. Due to the weak mechanical properties of the loess, this is stress-free to be distressed by the mining. A large number of mining ground fissures are generated on the gully slope. In addition, there is serious damage on the surface caused by rainwater erosion, leading to landslides, collapses, and other geological disasters. Therefore, the safety of people's lives, health, and property is endangered [2, 3]. For the problem of ground fissures on loess gully areas caused by coal seam mining, relevant scholars have studied the developing law and formation mechanism of ground fissures [4–6], the relationship model of mining-induced cracks and surface movement [7–9], and surface damage and prevention [10–12] using the methods of field measurements, numerical simulations, and theoretical analysis, and achieved rich results.

RETRACTED

Previous studies have generally simplified the gully terrain, which cannot reflect the real terrain. In addition, the overlying strata movement of coal seam and the evolution procedure of ground fractures and cracks are considered a problem of the discrete medium by means of intermittent huge deformation. However, the previously proposed methods cannot study the dynamic evolution law very well. Therefore, Itasca [13] proposed the theory of mesodiscrete element (which is also recognized as the theory of particle flow), namely the Particle Flow Code (PFC). An enormous amount of studies have proved that PFC is more suitable for studying the subsidence caused by coal seam mining. For example, Li and Wang [14] used the PFC2D simulation method to study the mine subsidence in the province of Shandong, China. They validated the practicability of using this method to simulate huge deformation. Similarly, the PFC2D approach was also used by Zhang et al. [15] to investigate the overlaying stratum movement and surface discontinuous deformation law in coal seam mining, and the viability of PFC on surface discontinuous deformation simulation was confirmed. The above research methods and results have important reference significance for the simulation study of mining-induced failure in the loess gully area. Therefore, we believe that there are research gaps for further investigation of the PFC in mining fields.

The objective of this paper is to provide the basis for the ecological restoration of land and the efficient and safe production of mines. In this paper, the numerical simulation and theoretical analysis methods are amalgamated to examine the overburden failure features and the evolution law of ground fissures in the loess gully area under different mining directions of the working face. The application of the method is illustrated on 8092 working faces of a mining area in the west of China. The results obtained from this research can provide useful information for deformation and failure prediction, working face mining method, and geological disaster assessment in the loess gully area. The following are the key and most important contributions of this study.

- The particle flow program is studied to examine and investigate the distortion and disaster procedure of overlying (covering or superimposed) rocks and surfaces in different mining directions on the loess gully area;
- The PFC program is then used to create a model of numerical calculation on complex loess gully area;
- A numerical calculation model under complex terrain conditions is established;
- We study the overburden failure characteristics and the evolution law of ground fissures in the loess gully area under different mining directions;
- The results obtained from this research can provide useful information for deformation and failure prediction, working face mining method, and geological disaster assessment in the loess gully area.

RETRACTED

The remaining of the paper is structured as follows. In Section 2, we provide a summary of the material, research methodologies, and procedures. Moreover, a review of the related work and state-of-the-art research contributions are also offered in this section. In Section 3, the simulation program and parameter calibration are discussed. Results are provided in Section 4. Discussion around the findings and results are elaborated in Section 5. We outline the major findings of this study along with limitations in Section 6. Lastly, Section 7 summarizes the outcomes of this paper along with several directions for future research.

## 2. Materials and Methods

### 2.1. Overview of Study Area

The terrain of a mining area in western China that fluctuates with a huge amount of gullies was developed. The surface of a typical loess gully area is covered by a thick loess layer. It should be noted that the dip length is approximately 127 m while the strike length of 8092 working face is approximately 400 m. In addition, the mining coal seam is 8 # coal seam. Moreover, the mining depth varies between 170–250 m, and the average thickness of the coal is 8 m. Similarly, the average dip angle of the coal seam is 6°. The roof of the working face is siltstone, 12 m thick, and the bottom plate is siltstone, 30 m thick. The top coal caving is completely automated, and the long-wall backward mining method is used on the working face. The ceiling is managed using all caving methods, and the mining progress is roughly 2.5 m/d.

A gully is across the working face area, as shown in Figure 1. The eastern slope is relatively slow with an average slope of 18°, and the western slope is relatively steep with an average slope of 24°. The profile of the gully is a “bowl” in shape, and the maximum drop between the top and bottom of the slope is about 75 m. Along with the continuous underground mining, the overlying rock in the gully area will move and deform, resulting in surface subsidence and failure. According to the survey results, there are many cracks on the slope surface. The crack width is about 0.1–0.2 m. There are obvious step cracks on the top and bottom of the slope [16]. The horizontal opening and vertical dislocation are large, which extremely distress the environmental setting (the surface cracks as shown in Figure 2). Therefore, the deformation and failure of the slope body in different mining directions are completely different.

RETRACTED

### 2.2. Deformation Characteristics of Mining Gully Area

The destruction process of the mining-induced gully area is usually from bottom to top. However, after coal seam mining, the superimposing strata endures collapsing towards the goaf, which breaks the original stress balance state. Moreover, the mining influence is gradually transferred from the goaf to the upward. Subsequently, the overburden deformation passed to the surface, and the slope above the goaf mainly moved vertically downward. The slope on both sides of the goaf moved closer to the center, affected by the sliding and mining action of the goaf face. Due to complex changes in the stress and displacement in the overburden, in fact, the tensile cracks were formed on the surface and extended along with the coal mining.

After the coal seam is mined to a certain area, different areas of the gully show different deformation characteristics due to locations. Therefore, according to the deformation characteristics, the study area is divided into five parts, which are shown in Figure 3. Area 1 is the strata above the goaf. The deformation is mainly vertical subsidence, and the horizontal deformation is small. Area 2 is the floor rock mass, which there will be an uplift arising. This is due to the fact that when the abutment pressure acting on the coal seam floor reaches or exceeds the critical value, then the floor rock mass will undergo plastic deformation and develop a plastic zone. With the increasing abutment pressure on floor rock mass, the plastic zone is connected into a piece and the floor is uplifted when reaching the maximum load of rock mass failure. Area 3 is the overburden outside the surface movement angle of goaf, which is basically not affected by mining. This is mainly affected by surrounding rock compressive stress, so the deformation is small.

Moreover, Area 4 is the overlying rock on both sides of the goaf, which is subjected to compressive stress in the vertical direction and tensile stress in the horizontal direction. Therefore, it dumps towards the epicenter of the goaf, and the right area of the goaf has a large range of horizontal movement due to the influence of slope sliding. Finally, Area 5 is below the slope, which is affected by the vertical compressive stress and the extrusion pressure of the rock mass on both sides. The deformation is mainly bending subsidence and affected by the slope slip. The maximum subsidence point is near the bottom of the gully [17–19].

RETRACTED

### 2.3. Simulations Using the Particle Flow Code (PFC)

The particle flow code (PFC) is a discrete element program and is quite changed from those techniques, which are based on the continuum mechanics methodology. In fact, the particle flow theory links both the macroscopic and microscopic mechanical features of elements and subsequently reflects the macroscopic position and status of elements over the process of contact and interaction. As a result, unlike the finite element method, PFC does not use a grid or grid concept [13]. The particle flow theory forms an arbitrary combination by connecting two or more particles. The force-displacement law and Newton's second law are used to simulate the block motion alternately.  Figure 4 describes the calculation cycle process [20]. In subsequent subsections, we briefly introduce the law of force-displacement and law of motion that basically form the particle flow code.

#### 2.3.1. Law of Force-Displacement

The particle flow program PFC2D/3D includes two types of contact, namely, (a) the particles contact with walls and (b) the particles with each other. Both types of contact are shown in Figures 5(a) and 5(b), respectively.

In the above figure, *R*_A_, *R*_B_, and *R*_b_ denote the radius of particles A, B, and b, respectively. Similarly, *x*_*i*_^*A*^, *x*_*i*_^*B*^, and *x*_*i*_^*b*^ characterize the center position of particles A, B, and b, respectively. Moreover, *x*_*i*_^*C*^ denotes the center position of the overlapping area in the contact, *d*_1_ represents the distance between centers of particles, *d*_2_ denotes the distance between Particle Center and Wall, *U*_n1_ is the amount of overlap between two particles, and *U*_n2_ is the amount of overlap between particle and wall, respectively.

(a) *Particle Contact with Each Other*. The distance between the centers of two particles *x*^*A*^ and *x*^*B*^ is characterized as *d*_1_ and is given by the following:
  (1) $$\begin{array}{c} d_{1}=\left|x_{i}^{A}-x_{i}^{B}\right|=\sqrt{{\left(x_{i}^{A}-x_{i}^{B}\right)}^{2}}. \end{array}$$
The overlap between the two particles *U*_n1_ is formulated as given by the following:
  (2) $$\begin{array}{c} U_{n1}=R_{A}+R_{B}-d_{1}. \end{array}$$
When *U*_n1_ > 0, it means that particles contact each other and they are in a state of compression. However, when *U*_n1_ < 0, it means that there is no contact between particles, and the particles are in a tensile state.
(b) *Particle Contact with Wall*. This should be noted that *d*_2_ is the distance between the particle center and the wall and can be computed as given by the following:
  (3) $$\begin{array}{c} d_{2}=\left|x_{i}^{c}-x_{i}^{b}\right|=\sqrt{{\left(x_{i}^{c}-x_{i}^{b}\right)}^{2}}. \end{array}$$
The amount of overlap between the particle and the wall *U*_n2_ is as follows:
  (4) $$\begin{array}{c} U_{n2}=R_{b}-d_{2}. \end{array}$$
When *U*_n2_ > 0, then it means that the particles contact with the wall and are under pressure. However, when *U*_n2_ < 0, then it means that there is no contact between the particles and the wall, and they are in a tensile state.

RETRACTED

#### 2.3.2. Law of Motion

This should be noted that in this paper, the single particle in the numerical calculation model is studied. Assuming that it is a rigid body, under the action of external force:

(5) $$\begin{array}{c} F_{i}=m\left(\overset{••}{x_{i}}-g_{i}\right), \end{array}$$

where *F*_i_ is the external force of the particle, *m* is the particle mass, $\overset{••}{x_{i}}$ is the particle accelerated speed, and *g*_*i*_ is the particle gravity accelerated speed. When the particles rotate, the particle velocity is calculated by a time step Δ*t*:

(6) $$\begin{array}{c} \overset{•\left(t+\Delta t/2\right)}{x_{i}}=\overset{•\left(t-\Delta t/2\right)}{x_{i}}-\left(\frac{F_{i}^{\left(t\right)}}{m}+g_{i}\right)\Delta t. \end{array}$$

Equation (6) is the particle velocity at the end of the one-time step. Therefore, the relationship between the center coordinates of particles and time can be obtained using the following:

(7) $$\begin{array}{c} \overset{\left(t+\Delta t/2\right)}{x_{i}}=x_{i}^{t}+\overset{•\left(t+\Delta t/2\right)}{x_{i}}\Delta t, \end{array}$$

where *t* denotes the time and *x* represents the particle. In contrast to standard numerical modeling methods, the PFC model is largely conquered and ruled by the microscopic characteristics of particles, which can accurately simulate the process of dynamic evolution in cracks. Therefore, it is necessary to assume that the particle unit is a rigid body, and the area of contact and communication between each other is trivial and overlaps [20].

## 3. Simulation Program and Parameter Calibration

### 3.1. Simulation Program

According to the actual field situation and drilling data (as shown in Figure 6), a two-dimensional 864 × 288 m^2^ particle flow mining field model was established based on the geological section of line A (refer to Figure 1) to simulate the coal seam beside the strike mining, as presented in Figure 6. The model has a total of 229,193 particles. Moreover, the overlying strata are layered, and the coal seam with particles was deleted in the mining simulation. In the calculation process of the proposed model, the vertical movement of the left and right boundary was allowed [21]. However, the horizontal lateral displacement was restricted as the PFC has a huge number of particles and the calculation is huge. As for the lower boundary, the horizontal movement was allowed, but the vertical displacement was restrained. The upper edge is a free borderline, which is loaded on the model using the law of gravity (the gravity acceleration is 9.8 m/s^2^).

RETRACTED

Since the working face is 400 m long, in order to simulate different underground mining directions, the open-off cut is at 243 m on the left boundary of the model and pushed forward 20 m each time to simulate the back slope mining. The open-off cut is at 221 m on the right boundary of the model, advancing 20 m each time to simulate the alongslope mining, as shown in Figure 7. After each excavation, the average ratio of the unbalanced force of the numerical model is less than or equal to 1e^−5^ considered balanced.

### 3.2. Parameter Calibration

A huge amount of studies have presented that the uniform joint model is, in fact, more appropriate for investigating the mechanical properties of rocks [22, 23]. In fact, this study also deals with the mechanical characteristics of rocks. As a result, the flat joint model describes the numerical computation model used in this study. The “trial-and-error approach” is used to calibrate the microscopic factors and limits of the particle flow model. The following are the particular measures to take. We can describe the proposed description of the measurement into two different stages that lead to parameter determination. We begin with a uniaxial compression test of numerical modeling of soil and rock in the first phase. The model's microscopic parameters are then adjusted in the second step to match indoor experimental findings with numerical simulation results. In this way, appropriate parameters for the proposed model may be determined. The microscopic characteristics of rock mass calibration in different layers are shown in Table 1.

## 4. Simulations and Results

### 4.1. Comparative Analysis of Caving Failure of Overburden Rock

The damage of the overburdened rock varied in different mining directions of the working face affected by mining, as shown in Figure 8. We discuss the comparative study in terms of (i) back slope mining; and (ii) along slope mining. The entire discussion in later sections is based on these two mining conditions.

RETRACTED

#### 4.1.1. Back Slope Mining

As soon as the working face advanced to 80 m, the primary collapse of the direct roof happened, and the collapse height was approximately 14.4 m. At this time, the bottom of the gully (front of the slope) was damaged by tensile stress in the subsidence area. As the working face continued to advance, the direct roof fell with the mining, and the goaf area increased gradually. When advancing to 100 m, the direct roof collapsed periodically, and the step distance of the periodic collapse was 20 m. As soon as the working face advanced to 140 m (the bottom of the gully), the rocks' blocks of the superimposing strata were crumpled unceasingly and occupied the goaf. In fact, this is due to the load of the loess layer. Moreover, the direct roof completely collapsed to the coal seam floor [24]. At this time, the failure range of the overlying strata was arched upward, and the slope was pulled by the soil in front of the tensile cracks. When advancing to 220 m, the overlying rock in the middle of the caving zone was compacted, and the cracks at the bottom of the gully were connected with the working face, forming a cut-through mining crack.

We observed that the tensile stress on the upper part of the slope increased and obvious tensile cracks appeared on the top of the slope (the trailing edge of the slope) due to tractive efforts of the middle and lower soil. At the end of the working face mining, the cracks on the top of the slope extended downward. Therefore, the slope was unstable with a downward sliding trend. There was a failure in the shape of a positive step on the surface. According to the simulation results, the gully area experienced the process of bottom crack failure, slope traction failure, and slope top sliding failure when the back slope was mined. The bottom crack was connected with the working face, and the failure mode was traction failure.

#### 4.1.2. Along Slope Mining

As soon as the working face advanced to 60 m, the immediate roof collapsed, and the collapse height was approximately 15.9 m. At this time, the slope crest sank underneath the effect of mining. In addition, the tensile force generated by the subsidence of the goaf is easy to make the slope crest push the slope body. However, there was no crack due to the large buried depth. When advancing to 80 m, the direct roof collapsed periodically, and the step distance of periodic collapse was 20 m. At this time, there were obvious cracks appearing at the bottom of the gully (front edge of the slope). With the further extension of the excavation range, the buried depth of the coal seam gradually decreased, and the failure range of the overlying rock was arched upward. The slope was pushed by the top of the slope and gradually inclined to the inside of the slope. When advancing to 140 m, tensile cracks opposite the slope aspect was generated at the top of the slope (the trailing edge of the slope). When pushing forward to 300 m, the middle overlying rock was completely compacted, and the cracks on the top of the slope continued to develop, further.

RETRACTED

In fact, the cracks at the bottom of the ditch were connected with the rock cracks formed in the goaf, and there were negative steps due to the pushing effect. After the mining of the working face, there was no obvious crack on the slope surface, and the bottom of the gully was seriously damaged. According to the simulation results, when mining the along slope, the gully area experienced the process of slope top subsidence pushing, gully bottom tensile failure, and slope top tensile failure. It should be noted that the gully bottom cracks were connected with the working face, and the failure mode was pushing failure.

Through the above analysis, it can be seen that whether along slope mining or back slope mining, the range of overburden failure in the loess gully area developed in arch upward. Moreover, we observed that the cracks at the bottom of the gully reached the slope after mining. When mining along slope, due to the decrease of buried depth and a step distance of the initial caving, there were obvious cracks at both, i.e., the top and bottom of the slope. As for the back slope mining, the disturbance near the slope surface was obvious and clearly visible, and there were obvious cracks appearing on the top, bottom, and surface of the slope.

This should be noted that previous scholars, such as Li et al. [11], also used a similar simulation experiment to study the slope stability under different mining directions. The authors demonstrated that the disturbance degree of the coal mining on the rock and soil near slope surface in back slope mining was significantly greater than that in the along slope mining. Their obtained results show that the numerical calculation was consistent with the simulation results of similar materials. In fact, this consistency is a positive symbol indicating that it is credible and correct for the PFC numerical simulation software on overburden failure and surface movement and deformation caused by underground coal mining.

The underground coal seam mining will cause stress redistribution around the goaf; therefore, the stope stress change can directly reflect the dynamic evolution of the overburden structure.  Figure 9 demonstrates the connection between the supporting pressure and the coal seam of different mining distances in different mining directions of the working face. It should be noted that the circle measured is on the floor of the coal seam, and the layout starts from the left side of the numerical model. The abutment pressure increase region is at the front and back of the goaf. We also observed that the tensile stress rise area is largely above the goaf, as can be seen in Figure 9. Furthermore, we observed that the main roof's initial collapse is backward, and the sustaining tension of the overlaying rock above goaf changes in a more complicated way than in the coal body. In addition, the peak supporting pressure values in the front and rear of the goaf gradually increase in line with the uninterrupted progression of the working face. After the along slope mining, the maximum supporting pressure of the monitoring point is approximately 10.66 MPa. At the end of the back slope mining, the peak supporting pressure of the monitoring point was observed as equal to 8.57 MPa; therefore, indicating that the supporting pressure above the coal pillar caused by slope mining changes significantly.

RETRACTED

### 4.2. Comparative Analysis of Cracks

In dissimilar mining directions of the working face, we observed that the deformation and failure of the loess gully area were significantly different. In the case of back slope mining, the bottom of the gully was first affected by mining, and then the moving deformation developed from bottom to top along the slope. The slope was mainly influenced by tractive efforts. In the case of along slope mining, the top of the slope was first affected by mining, and then the moving deformation developed from top to bottom along the slope. We observed during the numerical simulations that the slope was mainly impacted by the pushing efforts.

It can be seen in Figure 10 that there were three obvious cracks on the surface during the along slope mining. The cracks mainly existed at the bottom of the gully and the top of the slope. The cracks on the top of the slope were negative, and the width of crack a3 was 4.38 m. The cracks at the bottom of the gully were connected with the working face, and there were no obvious cracks appearing on slope surface. During the back slope mining, there were five obvious cracks on surface. The cracks mainly existed at the bottom of the gully, the slope surface, and the top of the slope. The cracks at the bottom of the slope were positive cracks, and the width of the crack i4 was 1.17 m. The cracks at the bottom of the gully were connected with the working face, and two obvious cracks appeared on slope surface. In general, the bottom of the gully was damaged seriously in both situations, i.e., when along slope mining and back slope mining. Moreover, the excavation of the coal seam in the direction of along slope has relatively small influence on the slope surface. However, it has a great influence on the flat ground of the slope.

RETRACTED

### 4.3. Comparative Analysis of Overburden and Surface Movement Deformation

The coal seam archaeological site will essentially cause deformation, displacement, and failure of covering and superimposing strata. In Figure 11, we have sketched the distribution of both the horizontal and the vertical displacement fields of the overlying or superimposing strata at the end of the first immediate roof caving and working face mining. In different mining directions of the working face, we observed that the first caving of the direct roof is significantly affected by horizontal stress and self-weight. In fact, this is due to tiny excavation space and displacement of the rock layer. However, as the working face advanced, then the covering strata continued to fill the goaf. We observed that the goaf was filled from the bending subsidence zone, fracture zone, and caving zone in a top to bottom approach. The fracture zone developed to the surface and formed mining cracks. At the end of working face mining, under the condition of back slope mining, the movement direction of the left slope was the same with goaf overburden, while the along slope mining was the opposite. Finally, the slope on both sides of the gully area was mainly horizontal displacement, and the bottom of the gully was mainly vertical displacement.

The displacement curve was drawn according to the displacement data of monitoring points at different positions on the surface.  Figure 12 is the surface subsidence curves corresponding to the initial collapse of the direct roof and at the end of the mining of working face for back slope mining and along slope mining. In different mining directions of the working face, with the extension of the mining range of the working face, the surface subsidence and influence range gradually increased. It should be noted that all surface subsidence curves were in a “U” shape, and the maximum subsidence point was near the bottom of the gully. The curve of subsidence was not symmetrical to the midpoint of the goaf. Moreover, the value of subsidence at the bottom of the gully was larger than that at other places. The maximum subsidence was observed at approximately 9.03 m in the case of the along slope mining, while the maximum subsidence was observed at 9.02 m in the case of the back slope mining. In fact, the subsidence is basically the same, therefore, this observation indicates that the advancing direction of the working face had no significant difference in the subsidence of the loess gully area with the same coal thickness.

RETRACTED

Figure 13 is the surface horizontal movement curve corresponding to the initial collapse of the direct roof and at the end of the working face mining for the back slope mining and the slope mining. Along with the working face advancing, the horizontal displacement of the surface and the influence range of the surface gradually increased, and the two extreme values moved to the edge of the basin. The surface horizontal movement curve showed a nonasymmetric state at zero point. In addition, affected by the slip of the gully slope, the surface horizontal movement value and influence range in the along slope direction were larger than those in the back slope direction. The maximum horizontal displacement was approximately 4.84 m for the along slope mining and approximately 4.17 m for the back slope mining. Subsequently, this indicates that the horizontal displacement caused by the along slope mining was significantly larger than that caused by the back slope mining.

## 5. Discussion

In this paper, the PFC is used to establish a numerical calculation model on a complex loess gully area and applied to the 8092 working faces in a mining area. Based on the analysis of the deformation and failure characteristics on the overlying strata soil of the goaf, it is concluded that the failure mode of the mining slope is highly correlated with the mining direction and relative position of the working face. In different mining directions of the working face, we observed that there is a difference in failure modes in the loess gully area. Therefore, according to the advancing direction of the working face, the failure mode of the loess gully area under the mining effect of a thick coal seam can be divided into the following two categories.

### 5.1. Back Slope Advancing Failure Mode

The advancing direction of the working face is opposite to that of the slope, and the coal seam starts to advance from the bottom of the gully. The destruction process can be divided into three independent stages:

1. In the primary phase of the working face mining, the covering and superimposing strata in the goaf sink due to self-gravity, and the slope on both sides of the gully moves into the goaf inside. Under the tensile stress of rock and soil in goaf, cracks first appear at the bottom of the ditch, as shown in Figure 14(a).
2. When the working face advances below the slope, the subsidence at the bottom of the ditch sinks even further. The tensile stress at the bottom of the ditch increases, and the cracks continue to extend. The mining effect extends from the bottom of the gully to the slope. There are tensile cracks appearing on soil mass due to tractive efforts of the front rock, as shown in Figure 14(b).
3. As the working face carries on to progress, then the scope of the mined-out area increases. The upper slope moved towards the free surface by the tractive effort of the lower slope, and there are tensile cracks appearing on the top of the slope. After the mining of the working face, the cracks at the bottom of the gully are connected with the mined-out area, forming connective cracks at the slope. The slope and cracks on the top of the slope extend continuously, as shown in Figure 14(c).

RETRACTED

### 5.2. Along Slope Advancing Failure Mode

In this mode, the advancing direction of the working face is the same as that of the slope, and the coal seam starts to advance from the top of the gully. The destruction process can be divided into three independent stages:

1. In the primary phase of the working face mining, the center of surface subsidence is at the top of the slope. The goaf causes essential variations of the inner stress within the covering and superimposing rocks, resulting in the subsidence behind the slope. Moreover, the top of the slope tends to move to the slope interior. There are no cracks formed due to the large burial depth of the coal seam, as shown in Figure 15(a).
2. When the working face advances to the middle and lower part of the slope, the center of surface subsidence transfers to the bottom of the slope. Moreover, the top of the slope inclines under the action of the goaf, resulting in the horizontal displacement pointing to the free surface. At this time, under the continuous action of the tensile force, there are obvious cracks at the bottom of the gully and the top of the slope, as shown in Figure 15(b).
3. With the uninterrupted improvement of the working face, the cracks at the bottom of the ditch and the top of the slope develop continuously. As the mining influence reaches a certain degree, the cracks will connect with the goaf and then form the connective cracks owing to the superficial suppressed deepness of the ditch bottom. The form of connective cracks is prevented owing to the large buried depth of slope crest, as shown in Figure 15(c).

## 6. Major Findings and Limitations

In this section, we briefly describe the contributions of this study and the major lessons learned from the experiments. We also list several limitations of our work that we aim to consider as part of the ongoing research.

RETRACTED

### 6.1. Major Contributions of This Study

In this study, we studied and used the particle flow program in order to explore and examine the distortion and disaster process of covering and superimposing rocks and surfaces in different mining directions in the loess gully area. Moreover, the numerical calculation model under complex terrain conditions was established. As a result, two kinds of slope deformation and failure modes under along slope mining and back slope mining were obtained, which provided a reference for the application of the particle flow method in this aspect, the deformation evaluation of mining-induced slope and ground protection.

### 6.2. Key Findings and Outcomes

The following are the key findings of our research that were observed during the experiments.

1. The failure range of overlying strata in the loess gully area is arched upward, whether the back slope mining or the along slope mining. During the back slope mining, we observed that the gully area experienced the process of bottom crack failure, slope traction failure, and slope top sliding failure. As for the along slope mining, we noticed that the gully area experienced the process of slope top subsidence pushing, gully bottom tensile failure, and slope top tensile failure.
2. When the back slope mining is adopted for the working face, cracks mainly exist at the bottom of the gully, the slope surface, and the top of the slope. For along slope mining, the cracks mainly exist at the bottom of the gully and the top of the slope. The bottom of the gully is damaged seriously when along slope mining and back slope mining. The slope surface was affected relatively in the excavation direction of the coal seam on along slope, but more on the upper slope. In order to ensure the stability of the slope, the along slope mining is better than the back slope mining.
3. In different mining directions of the working face, the surface subsidence takes on a consistent character with the horizontal movement. The maximum surface subsidence and horizontal movement caused by the back slope mining were found to be significantly less than those caused by the along slope mining. The maximum subsidence point and the zero value of the horizontal movement are inclined to the bottom of the gully due to the slip of the gully slope. Under the same mining conditions, we observed that the advancing direction of the working face has a slight difference in the subsidence of the loess gully area and greater on the horizontal movement.
4. The movement simulation of particles on the PFC is based on (a) the second law of Newton; (b) the law of force displacement, which might spontaneously show the process of dynamic evolution in terms of fracture development and overburden structure. The change in abutment stress above goaf is more complicated than that in the coal body, as evidenced by monitoring the abutment pressure above the coal pillar. Similarly, the change of abutment pressure above the coal pillar caused by the along slope mining is greater. The change of stope stress can directly reflect the dynamic evolution of the overburden structure.

RETRACTED

### 6.3. Limitations of This Study

The numerical model created by the PFC method is, in fact, made up of a large number of particles that require a lot of computation. For that reason, instead of the classical PFC, the PFC2D version is adopted in this study. In fact, the PFC2D has small computational calculations but comes at the cost of limitations. In this way, the change in the horizontal direction is not considered in the study of the deformation and failure law of the gully area. The future research direction will focus on the subsidence research of the three-dimensional mining area. Moreover, additional characteristics of rocks, parameters, and mining conditions should be taken into account.

## 7. Conclusions and Future Work

In this study, we used the particle flow program to examine the distortion and catastrophe process of the covering and superimposing rocks and surfaces in diverse mining directions on the loess gully area and the numerical calculation model under complex terrain conditions was established. Two kinds of slope deformation and failure modes under along slope mining and back slope mining were obtained, which provided a reference for the application of the particle flow method in this aspect, the deformation evaluation of mining-induced slope and ground protection. Based on the analysis of the distortion and disaster characteristics on the overlying strata soil of the goaf, it is concluded that the failure mode of the mining slope is highly correlated with the mining direction and relative position of the working face. This decreases possible jeopardies and tragedies that distress social well-being and health. Consequently, this guarantees developed welfare and safety from the perspective of healthcare in the field of geological mining.

In the future, the change in horizontal direction must be taken into account during the study of the deformation and failure law of the gully area. Since the PFC consists of a huge number of articles, therefore, it needs huge computational calculations. The future research direction will focus on the subsidence research of the three-dimensional mining area. Moreover, other methods, including machine learning and artificial intelligence, can be integrated into the proposed PFC-based model to improve its accuracy and performance. Moreover, in the future, we will investigate how the proposed model should be applied for the evaluation of landslide susceptibility in the coal mining subsidence areas.

RETRACTED

## Figures and Tables

**Figure 1:** Topography, i.e., gully across the working face area.

**Figure 2:** The surface cracks that affect the ecological environment.

**Figure 3:** Deformation characteristics of the mining gully area.

**Figure 4:** The process of calculation cycle for particle flow code (PFC).

**Figure 5:** Visual representation of the two types of contact. (a) Contact between particle with particle; (b) contact between particle with the wall.

**Figure 6:** Borehole histogram.

**Figure 7:** The particle flow field model.

**Figure 8:** Deformation and failure of overburden rock in various mining conditions; (a) back slope mining and (b) along slope mining.

**Figure 9:** The distribution of supporting pressure of simple roof through different propulsion distances and mining conditions.

**Figure 10:** Crack distribution diagram (a) back slope mining, and (b) along slope mining.

**Figure 11:** Horizontal and vertical displacements caused by back slope and along slope mining. (a) Vertical displacement (m) (b) horizontal displacement (m).

**Figure 12:** Subsidence curve.

**Figure 13:** Horizontal displacement curve.

**Figure 14:** Failure mode of the back slope mining.

**Figure 15:** Failure mode of the along slope mining.

**Table 1:** The microscopic characteristics of the rock strata.

Sign	Explanation	Loess layerS10	SandymudstoneS6, S8	Medium-coarsesandstone S5, S7	MudstoneS4, S9	Coal S2	SiltstoneS1, S3
*γ* (KN/m^3^)	Volume-weight	18	24	25	24	16	24
*R* (cm)	Minimum radius of particles	40	40	40	40	40	40
*R*_max_/*R*_min_	Particle radius ratio	1.6	1.6	1.6	1.6	1.6	1.6
*E* ^*∗*^(GPa)	Effective modulus of flat joint	0.4	14.2	22	13.5	4	28.2
*K* ^*∗*^	Rigidity ratio of flat joint	2	2	2	2	2	2
*σ*_*c*_ (MPa)	Average tensile strength of flat joint/standard deviation	0.1/0.025	0.8/0.2	1/0.25	0.8/0.2	0.25/0.0625	1.2/0.3
C (MPa)	Average cohesion of flat joint/standard deviation	4/1	20/5	20/5	20/5	10/2.5	20/5

## Data Availability

The raw/processed data required to reproduce these findings cannot be shared at this time as the data also form part of an ongoing study.
